# Recent Progress of Chronic Stress in the Development of Atherosclerosis

**DOI:** 10.1155/2022/4121173

**Published:** 2022-03-08

**Authors:** Shang Gao, Xiang Wang, Ling-bing Meng, Yuan-meng Zhang, Yue Luo, Tao Gong, De-ping Liu, Zuo-guan Chen, Yong-jun Li

**Affiliations:** ^1^Department of Vascular Surgery, Beijing Hospital, National Center of Gerontology, Institute of Geriatric Medicine, Chinese Academy of Medical Sciences, No. 1 DaHua Road, Dong Dan, Beijing 100730, China; ^2^Graduate School of Peking Union Medical College and Chinese Academy of Medical Sciences, No. 9 Dongdansantiao, Dongcheng District, Beijing 100730, China; ^3^Department of Cardiology, Beijing Hospital, National Center of Gerontology, Institute of Geriatric Medicine, Chinese Academy of Medical Sciences, No. 1 DaHua Road, Dong Dan, Beijing 100730, China; ^4^Department of Internal Medicine, The Third Medical Centre of Chinese PLA General Hospital, The Training Site for Postgraduate of Jinzhou Medical University, Beijing, China; ^5^Department of Respiratory, The First Affiliated Hospital of Jinzhou Medical University, Jinzhou, Liaoning 121001, China; ^6^Department of Neurology, Beijing Hospital, National Center of Gerontology, Institute of Geriatric Medicine, Chinese Academy of Medical Sciences, No. 1 DaHua Road, Dong Dan, Beijing 100730, China

## Abstract

With the development of the times, cardiovascular diseases have become the biggest cause of death in the global aging society, causing a serious social burden. Atherosclerosis is a chronic inflammatory disease, which can occur in large and medium-sized blood vessels in the whole body. It takes atherosclerotic plaque as the typical pathological change and endothelial injury as the core pathophysiological mechanism. It is the pathological basis of coronary heart disease, peripheral artery disease, cerebrovascular disease, and other diseases. Recent studies have shown that chronic stress plays an important role in the occurrence and development of atherosclerosis, endothelial injury, lipid metabolism, and chronic inflammation. This process involves a large number of molecular targets. It is usually the cause of atherosclerotic cardiovascular and cerebrovascular diseases. If chronic stress factors exist for a long time, patients have genetic susceptibility, and the combination of environmental factors triggers the pathogenesis, which may eventually lead to complete blockage of the blood vessels, unstable rupture of plaques, and serious adverse cardiovascular events. This paper reviews the role of chronic stress in the occurrence and development of atherosclerosis, focusing on the pathophysiological mechanism.

## 1. Introduction

With the development of economy, the total prevalence of cardiovascular disease in the world is increasing year by year. At present, the total number of cardiovascular diseases exceeds 587 million. In 2019 alone, 18.6 million people died and 34.4 million were disabled, with an upward trend year by year [1]. Among them, atherosclerosis is the pathological basis of a variety of cardiovascular and cerebrovascular diseases, which is easy to appear in various diameter arteries, common in the coronary artery, aorta, carotid artery, etc. [2]. It is generally believed that atherosclerosis originates from various stimulating factors, including mechanical factors, LDL particle deposition, toxins, and viruses, which lead to the destruction of endothelial cells on the arterial intima. The damaged endothelial cells secrete cytokines and growth factors, attract monocytes gathering, migrate to endothelial cells, and transform into macrophages, These macrophages swallow cholesterol-rich oxidized low-density lipoprotein (ox LDL) through TLRs to form foam cells [3]. The persistence of proinflammatory factors leads to the accumulation of more macrophages, mast cells, and activated T cells and B cells into foam cells, showing a lipid streak [4]. At the same time, growth factor activates smooth muscle cells in the arterial membrane, enters the intima and secretes extracellular matrix, makes the endothelium thickening, fibrosis, and hardening, and absorbs lipids through LPL receptors to form foam cells [5, 6]. The two types of foam cells are progressed and eventually become atherosclerotic.

Chronic stress refers to the nonspecific pathophysiological response caused by the change of the body's steady state under the long-term stimulation of various adverse factors in vivo and abroad. Generally speaking, it is the emotional experience of people under the pressure that they are difficult to adapt [7, 8]. The source of this stress is often psychological stress. It is generally believed that there will be feelings of tension, depression, and sadness under psychological stress; the sources of this stress are often four categories: work, family, finance, and major life events. A large cohort study of more than 10000 people found that one or more levels of psychological stress in patients with myocardial infarction were significantly elevated [9]. For the animal model of chronic stress, the commonly used chronic stressors include fasting, closed environment, long-term forced swimming, or electrical stimulation. Chronic stress is one of the promoting factors of many peripheral vascular diseases. Studies have shown that chronic stress can cause a variety of cardiovascular diseases, such as dysfunction of vascular smooth muscle cells, even leading to rupture of aortic aneurysm [10, 11]. The most important thing is that chronic stress can cause the occurrence and development of atherosclerosis. Studies have shown that chronic stress is an independent risk factor for carotid atherosclerosis in Mexican women [12]. For the rat model of atherosclerotic intimal hyperplasia, most carotid arteries are blocked by atherosclerotic lesions after two weeks under chronic stress [13]. The possible pathophysiological mechanism of promoting the progression of atherosclerosis involves many aspects. Chronic stress reduces the activity of hypothalamic pituitary adrenal axis, leads to the decline of anti-inflammatory ability, stimulates the sympathetic adrenal medulla, and increases the content of blood catecholamine. Catecholamine binds to the *β*-adrenal receptor on the surface of macrophages, stimulates macrophages to produce more cytokine catecholamine, induces the expression of related inflammatory cytokines, and promotes the progress of inflammation [14–16]. Chronic stress can also promote oxidative stress and vascular sensitivity by increasing blood triglycerides and low-density lipoprotein. It can also reduce the content of NO synthase and NO, which can produce contractile effect on the aortic vessels and promote the development of atherosclerosis [17, 18]. Chronic stress can also lead to changes in plaque stability and poor prognosis of atherosclerosis.

The purpose of this paper is to comprehensively review the effects of chronic stress on the occurrence and development of atherosclerosis, pay special attention to the pathophysiological mechanism of chronic stress in the occurrence and development of atherosclerosis, and especially explore how chronic stress accelerates the progress of atherosclerosis from the aspects of chronic inflammation, hemodynamics, lipid metabolism, adipose tissue interaction, and the progress of atherosclerotic plaque, so as to provide some ideas for clinical intervention and basic research (Figure 1).

### 1.1. Inflammation: The Core Cause Induced by Chronic Stress

It has been elucidated that atherosclerosis is essentially a chronic inflammatory disease. Inflammation plays a role in all stages of atherosclerosis, including accumulation of foam cells, formation of fatty streaks and fibrous plaques, rupture of acute plaques, and formation of thrombus [19–23], eventually leading to atherosclerosis and thrombotic complications. A large number of studies have confirmed that for chronic stress, it is currently considered that it may lead to chronic low-grade inflammation through a variety of ways and is related to atherosclerosis. Inflammation is even further developed by activating platelets and endothelial dysfunction, which is reviewed in detail in the part of endothelial dysfunction.

Clinical and animal experiments have shown that for inflammatory factors, long-term chronic stress can increase the concentration of blood cortisol through HPA axis on the one hand and change the steady-state balance of autonomic nervous system and increase the content of catecholamine by stimulating sympathetic adrenal system and reducing the vagus nerve tension on the other hand. Both cause the decrease of anti-inflammatory ability; the continuous progress of inflammation; the increase of the concentration of inflammatory cytokines, serum IL-6, and TNF; the increase of the expression of IL-6 and TNF in the liver and spleen; and the increase of CRP can also cause the change of inflammatory cytokines [24–26]. In addition, norepinephrine (NE) and neuropeptide Y (NPY) released by activated sympathetic activity can also promote the phosphorylation of mitogen-activated protein kinase (MAPK) or the release of high-mobility group protein B1 (HMGB1), thus inducing systemic inflammation and accelerating the development of cardiovascular diseases [27]. In addition, chronic stress can also enhance the activity of dipeptidyl peptidase-4 (DPP4) in plasma and reduce the concentration of plasma glucagon-like peptide (GLP-1) and adiponectin (APN), so as to promote the development of inflammation [28, 29]. However, it is still unclear whether it is possible to reduce the promoting effect of chronic stress on atherosclerosis by targeted inhibition of cellular inflammatory factors. For inflammatory cells, chronic stress can cause bone marrow cells to enter a highly reactive inflammatory state, cause leukocyte proliferation, and increase the number of circulating inflammatory monocytes [30, 31]. In addition, inflammatory cells and inflammatory cytokines are not isolated from each other. The activated sympathetic adrenal system can increase the number of immune response cells expressing M receptor and inflammatory cytokines [32, 33] and produce a large number of cytokines. After HPA axis changes caused by chronic stress, TLR4/NF-*κ*B pathway activates proinflammatory cytokines such as MCP-1 and IL-1*α*and IL-6 and, at the same time, leads to the increase of intimal macrophage/monocyte ratio [17, 34], so that under the interaction of inflammatory factors and cells, endothelial homeostasis changes and inflammation further progresses and forms a vicious circle [35]. Interestingly, recent studies have also demonstrated that TLR4/NF-*κ*B pathway also downregulates HMGB1 protein-mediated PPAR*γ*/LXR*α*. The expression of ABCA1 pathway reduces the antiatherosclerotic effect of ATP binding cassette transporter 1 (ABCA-1) [36]. Therefore, the progression of atherosclerotic inflammation caused by chronic stress is a complex system, and the specific mechanism needs to be further studied.

## 2. Results and Discussion

### 2.1. Dyslipidemia: An Important Risk Factor of Chronic Stress Promoting the Progression of AS

Dyslipidemia is the first recognized independent risk factor for intima and media thickening of atherosclerosis [4]. Higher levels of serum low-density lipoprotein and total cholesterol can induce atherosclerotic precipitation, while low-density lipoprotein oxidation modified product (ox LDL) can be recognized and ingested by monocyte macrophage TLR and finally form lipid plaque [37]. However, simple dyslipidemia cannot fully explain the progress of atherosclerosis. Some studies have conducted large-scale clinical trials with statins that can reduce low-density lipoprotein, and cardiovascular events have been significantly reduced. However, even with intensive statin therapy, the ability to prevent cardiovascular events is still limited to 30% to 40% of treated patients [38], indicating that hyperlipidemia is not the only cause of atherosclerosis. Therefore, chronic stress comes into our sight. It has been reported that it can induce hyperlipidemia and lipid oxidation, cause lipid deposition to form plaque, may also lead to hypercoagulable state of arterial thrombosis, accelerate the progress of atherosclerosis, and produce adverse results [39, 40].On the one hand, it has been reported that in the control study of stressed mice and ordinary mice, high concentrations of serum total cholesterol, triglycerides, low-density lipoprotein, and very low-density lipoprotein can increase the atherosclerosis index of the chronic stress group, while the change of mice in the control group is not obvious [37]. In turn, chronic stress will change the blood lipid profile. In the study of hyperlipidemia rabbit model, with the extension of chronic stress exposure, the circulating concentrations of cholesterol, LDL, VLDL, and TG will significantly increase with time, while high-density lipoprotein will remain unchanged or decrease, and the atherosclerosis index will increase [18, 40, 41].

Hyperlipidemia and chronic stress interact to form a vicious circle, which together leads to the progress of atherosclerosis. Some researchers stimulated mice with chronic mild unpredictable stress (CMS), which also proved that CMS can increase the plasma concentration of corticosterone and lipids, increase the atherosclerosis index, and lead to the impairment of thoracic aortic function [42]. In addition, some studies stimulated atherosclerotic mice with cold stress, and the blood lipid of stressed rats was significantly higher than that of the control mice. Pathologically, it was found that cardiac oxidative stress was aggravated, macrophage infiltration and proinflammatory gene expression were found in the left ventricle and visceral adipose tissue, and the incidence of cardiac-related adverse events was further increased [43]. From the perspective of mechanism, chronic stress for more than 4 weeks can cause adrenal cortical stress hyperplasia; increase GC synthase, citrate synthase, and ketoglutarate dehydrogenase; increase glucocorticoid; promote ATP synthesis and energy metabolism [40, 44]; appear insulin resistant; promote hepatic triglyceride synthesis; and delay the binding and degradation of LDL by hepatocytes. Finally, it promotes circulating hyperlipidemia, which will continue after the removal of chronic stressors [45–47]. Chronic stress can also induce adrenoceptor desensitization and receptor downregulation in adipocytes, resulting in reduced catecholamine-induced lipolysis capacity and lipid accumulation [48]. In addition, it has been studied that the fatty acids released by lipolysis of adipose tissue under chronic stress can be used as substrates for cholesterol synthesis, causing the increase of blood cholesterol and aggravating the progress of atherosclerosis [49]. In addition, chronic stress beyond the threshold will stimulate the sympathetic nerve to directly upregulate the expression of neuropeptide Y or indirectly upregulate the expression of neuropeptide Y and its receptor Y2R by increasing glucocorticoid, resulting in abnormal lipid metabolism [50]. It can also regulate ABCG1 gene by upregulating TLR4, mediating inflammation and intracellular lipid accumulation are also necessary ways for macrophages to transform into foam cells [51–53]. In addition, the expression of aortic matrix metalloproteinase -9 (MMP-9) and MMP-2 gene will also increase, reduce the expression of adiponectin in preadipocytes, promote LDL-induced monocyte uptake of lipids, and promote the formation of foam cells [28].

### 2.2. NO: The Core Molecule Causing Endothelial Dysfunction Under Chronic Stress

Normal endothelium maintains vascular tension and structure by regulating the balance between vasodilators (such as NO and prostacyclin) and vasoconstrictors (such as endothelin-1 and norepinephrine) [54].The result of endothelial dysfunction is to cause the progress of atherosclerosis, hypertension, and other changes. Among them, NO is an important vasodilator molecule, which cooperates with other endothelial-derived factors to participate in endothelium-dependent relaxation [55, 56]. NO is produced by the precursor L-arginine, which is affected by NO synthase, and at least three functional forms of NO synthase (endothelial (eNOS), neuronal (nNOS), and inducible (iNOS)) are known [57]. In terms of function, NO is related to various endothelial functions, including regulating vascular tension, platelet aggregation, and vascular smooth muscle cell proliferation [58].

The response of vascular endothelium to chronic stress is the adaptation to its harmful effects. This adaptation is NO dependent [59, 60]. In early chronic stress, chronic stress hormone reduces endothelial injury by stimulating the release of ET-1 and maintaining a high level of NO [61]. In the study of different types of chronic stress mouse models, it was found that the level of NOx increased significantly and the time-dependent iNOS activity increased [57]. This increased activity of NO system will weaken the vasoconstrictive effect of catecholamine and ANGII [62, 63] and platelet aggregation caused by increased sympathetic activity and resist the vascular system disorder caused by chronic stress [64, 65].It was also confirmed in another study. Early chronic stress will have vascular relaxation changes and reach the peak eight weeks after the administration of chronic stressor and decrease twelve weeks. However, the analysis of blood components found that this is related to the reduction of relaxation components independent of NO, and NO will not decrease in the early stage [28]. At the same time, early chronic stress can also improve the response of endothelium to NO, weaken the vasoconstriction caused by calcium ion, and play a certain role in vasodilation [66].

However, long-term chronic stress may lead to endothelial dysfunction, vascular remodeling, and systolic hypertension through vascular oxidative stress. The decrease of endothelium-dependent relaxation was observed in this process, which may be related to the decrease of endothelial NO synthase activity and the decrease of NO bioavailability [67, 68]. In terms of mechanism, excessive ROS is produced under chronic stress, which changes the balance of oxidants and antioxidants and leads to the development of various pathological states, dysfunction of intracellular mitochondria, interruption of energy pathway, and induction of apoptosis [69]. More importantly, it causes the reduction of NO production and disorder of vasoconstriction and relaxation and induces MMP-2 and MMP-9 to decompose fiber caps containing collagen, elastin, and proteoglycan. The removal of ROS can reduce blood pressure, which can also explain the harm of chronic stress [69–72], and these injuries are controlled by the differential regulation of NO [73]. Studies have shown that *Salvia miltiorrhiza* can restore endothelial function to a certain extent by increasing the amount of NO and the level of eNOS [72]. Similarly, the role of chronic stress may also involve NO-dependent endothelial dysfunction [28]. Studies have shown that there is a compensatory vasodilation mechanism in chronic stress mice with impaired NO bioavailability. This mechanism may be related to hydrogen peroxide as a compensatory dilation metabolite, which ensures vascular reactivity to a certain extent [68]. Similarly, after long-term chronic stress, the effect of related hormones can no longer be antagonized by vasodilators such as NO. For example, glucocorticoid and proinflammatory cytokines, norepinephrine, and endothelin-1 may aggravate endothelial dysfunction by reducing eNOS expression, increasing eNOS inactivation, and promoting NO degradation and antagonism of NO-induced vasodilation [74]. On the other hand, the elevation of aldosterone and sodium and water retention of glucocorticoid can hardly get NO against [75–77]. Therefore, many factors work together to cause hemodynamic decompensation after long-term chronic stress.

### 2.3. Adipose Tissue: Correlates under Chronic Stress

Obesity is associated with chronic stress and atherosclerosis. Chronic stress can cause excessive fat accumulation to a certain extent [43]. Studies have shown that obesity can increase the incidence rate of cardiovascular and cerebrovascular diseases. Obesity may cause inflammation and atherosclerosis by secreting a large number of adipokines and proinflammatory cytokines [78, 79]. But interestingly, through big data analysis, it can be found that there is no nonlinear relationship between the degree of obesity and atherosclerosis. Studies have shown that when CPC is used as an index of endogenous vascular proliferation to study this paradox, the number of good outcomes of high regenerative capacity (i.e., high CPC count) in obese people is more [80]. On the other hand, the degree of visceral obesity and BMI index is not linear [81]. Chronic stress promotes the accumulation of visceral fat. Therefore, there are some deficiencies in using BMI as a link between obesity, cardiovascular and cerebrovascular adverse events and chronic stress. Moreover, the expansion of aorta, slowing down the shear force of blood flow and playing the role of endothelial protection is also one of the reasons for the obesity paradox [82].

At present, chronic stress is more closely related to abdominal obesity. One view is that excessive glucocorticoid secretion caused by chronic stress will affect fat distribution and promote the selective accumulation of visceral fat [78], accompanied by a series of metabolic disorders, including dyslipidemia, impaired glucose tolerance and insulin resistance, and unstable or elevated blood pressure [83–86]. In addition, these factors are harmful to arteries and promote the development of atherosclerosis. However, the current research suggests that chronic stress has little to do with aggravating the inflammatory response of abdominal obesity and may increase the secretion of proinflammatory cytokines to a certain extent [87, 88].Some research evidence suggests that peripheral neuropeptide Y induced by chronic stress may play an important role [89]. It may also promote fat accumulation through a variety of stress behavior reactions, resulting in stronger cardiac sympathetic tension after obesity, exacerbate abnormal heart rate and metabolism, and increase the risk of cardiovascular disease [90]. Interestingly, the simultaneous occurrence of chronic stress and obesity is not necessarily a vicious circle. Some studies on mice have shown that high-fat diet can alleviate the anxiety caused by chronic stress and improve the activity intensity of anxious animals [91]. At the same time, the high-fat diet under chronic stress may also reduce the level of corticosterone and reduce the incidence of obesity to a certain extent [91, 92], but some studies have shown that various types of delicious food can also increase body weight [93].Therefore, understanding the lipid metabolism under stress is of great significance to study the relationship between chronic stress and atherosclerosis. In addition, a special type of adipose tissue, perivascular adipose tissue, plays an important role in the maintenance of vascular function. It secretes a large number of paracrine signal molecules, which affect the function of vascular wall through direct diffusion, trophoblast, or catheter [94]. However, chronic stress causes perivascular adipose tissue to become an inflammatory phenotype, which is characterized by changes in the spectrum of adipokines, cytokines, and chemokines, resulting in activation of arterial oxidative stress, reduction of NO bioavailability, reduction of EDD, and increase of aortic stiffness. From the perspective of mechanism, it may be related to the overactivation of sympathetic nervous system and the increase of aldosterone production [95, 96].

### 2.4. Plaque Progression: The Culprit of Adverse Events Caused by Chronic Stress

The latest research shows that chronic stress can not only cause the progression of atherosclerotic plaque but also accelerate the change of plaque instability. On the one hand, after 12 weeks of mild chronic stress exposure, the area of main atherosclerotic plaque in the ApoE-/-mice doubled compared with the unexposed mice [97]. On the other hand, in many studies on coronary artery, ascending aorta and abdominal aorta, histopathology shows that in the animal model of atherosclerosis, chronic stress can cause acute thrombosis and plaque instability. It is characterized by accelerated apoptosis, thinning of fiber cap, lipid deposition, increased macrophages and neovascularization, and increased degree of perivascular fibrosis, but the reduction of smooth muscle cells and intimal mediators such as type I collagen and elastic fibers especially significantly promotes the degeneration of the inner side of the plaque, which generally aggravates the inflammatory phenotype of atherosclerosis and makes the plaque easy to fall off from the vascular wall. Large-scale clinical cohort studies have shown that there is a causal relationship between mental changes caused by chronic stress and the progression of atherosclerosis and the decrease of plaque stability in people with coronary heart disease [98–101]. The reason can be found that chronic stress can aggravate the level of inflammation and oxidative stress through inflammatory cytokines, oxidized low-density lipoprotein, mechanical damage caused by elevated blood pressure and enhanced HPA axis function, resulting in the imbalance of vascular smooth muscle cell proliferation and apoptosis, and reduce the stability of plaque [98, 102]. Some studies used a multisystem 18F-FDG-PET/CT imaging. The results show that long-term elevated stress-related neurobiological activities will promote leukocyte production and inflammatory progression and then increase the plaque load of ARI and noncalcified coronary artery, resulting in reduced plaque stability [103]. Some studies have studied the proapoptotic effect of chronic stress at the molecular level. Chronic stress can increase the activity of DPP4 and decrease the expression of GLP-1 and cause the progression of plaque inflammation and aggravation of oxidative stress. At the same time, DPP4 inhibitor has certain therapeutic significance on endothelial injury and vascular aging, while exenatide, a GLP-1 analogue, decreased the expression of MMP-9 and MMP-2 genes in (ApoE-/-) mice. Stimulation of adiponectin expression in preadipocytes inhibited the formation of monocyte-derived foam cells induced by LDL, thereby slowing plaque progression [28, 29, 104]. High levels of cortisol induced by chronic stress can induce low levels of miRNA 25, increase proapoptotic proteins, induce apoptosis of smooth muscle cells, and reduce plaque stability. This effect is significantly related to the inhibition of targeting moap1 and P70S6K pathways [105]. In addition, chronic stress can promote the expression of cysteinyl cathepsin S (Cat-S), directly affect TLR2/4, cause the progression of inflammation and oxidative stress, proliferate vascular smooth muscle cells, lead to neointimal hyperplasia, and reduce plaque stability [106]. The absence of cysteinyl cathepsin K (Cat-K) prevents the development of experimental neointimal hyperplasia by weakening the excessive effect of inflammation, the production of oxidative stress, and the proliferation of VSMC, which has a synergistic effect with Cat-S [107]. It has been reported that chronic stress induces rapid intimal hyperplasia in angioplasty injured rats (i.e., animal model of intimal injury) through neuropeptide Y (NPY), which may be related to intimal hyperplasia and plaque progression of atherosclerotic nature [108]. The unstable progression of atherosclerotic plaque is also related to the immune environment. It has been reported that chronic stress can significantly affect the local immune environment of mouse aorta, cause the accumulation of inflammatory cells in plaque, and reduce its stability [109].

## 3. Conclusion and Prospect

With the change of life rhythm, the impact of chronic stress on human health has attracted more and more attention. We reviewed the effects of chronic stress on the occurrence and development of atherosclerosis, focusing on the pathophysiological mechanisms, including chronic inflammation, hemodynamic changes, lipid metabolism changes, adipose tissue interaction, plaque progression, and so on. The related changes will eventually lead to abnormal vascular structure and atherosclerotic cardiovascular disease. But due to a perfect self-regulation mechanism in the body, acute internal environment disorder has a relatively weak impact on program genes. However, under the condition of chronic stress, abnormal gene expression can be induced continuously. Since chronic stressors cannot be removed, gene-induced changes in abnormal cell function are irreversible. At present, it has been confirmed that atherosclerosis is a pathological state in which the apoptosis of endothelial cells is excessive and apoptosis of smooth muscle cells is insufficient. The abnormal expression of these cells is closely related to the disturbance of internal environment and endocrine function under chronic stress. The anti-inflammatory effect of statins is based on lipid regulation to reduce the decline of inflammatory factors caused by chronic stress in the body. Chronic diseases such as diabetes and hypertension can be used as chronic stressors to increase the corresponding inflammatory factors and promote the formation of atherosclerosis. Drugs (including betas, angiotensin-converting enzyme inhibitors, angiotensin receptor antagonists, *β*-blockers, and antiplatelet drugs) are essential in the treatment of these diseases and control the presence of corresponding chronic stress factors. In future studies, we will pay more attention to the influence mechanism of chronic stress on atherosclerosis, and it is a novel insight to develop targeted drugs for the prevention and treatment of atherosclerosis against chronic stress in the future.

## Figures and Tables

**Figure 1:** Flow diagram showing the procedure of searching the references in the databases.

## Data Availability

The data used to support the findings of this study are available from the corresponding author upon request.

## Abbreviations

ABCA-1: ATP-binding cassette transporter 1
ADAMTS7: A disintegrin and metalloproteinase with thrombospondin motifs 7
ANGPTL3: Angiopoietin-like protein
Apo A-I: Apolipoprotein A-I
Apo E: Apolipoprotein E
APN: Adiponectin
AVP: Vasopressin
ox LDL: Oxidized low-density lipoprotein
Cat-K: Cathepsin K
CRH: Corticosteroid-releasing hormone
CRP: C-reactive protein
CPC: Circulating progenitor cells
CS: Citrate synthase
DPP4: Dipeptidyl peptidase 4
GLP-1: Glucagon-like peptide-1
HMGB1: High-mobility group B-1
HPA: Hypothalamic pituitary adrenal axis
ICAM-1: Intercellular adhesion molecule-1
IL-1: Interleukin-1
IL-6: Interleukin-6
LPL: Lipoprteinlipase
LXR *α*: Recombinant liver X receptor alpha
MAPKs: Mitogen-activated protein kinases
MCP-1: Monocyte chemoattractant protein-1
MMP-9: Matrix metalloproteinase-9
NE: Noradrenaline
NF-*κ*B: Nuclear factor kappa-B
NPY: Nerve peptide Y
OGDC: Oxoglutarate dehydrogenase complex
PPAR-*γ*: Peroxisome proliferator-activated receptors-*γ*
RAAS: Renin-angiotensin-aldosterone system
TNF: Tumor necrosis factor
TLR4: Toll-like receptor 4
VSMC: Vascular smooth muscle cell.
